# An Overview of Deep Learning Techniques on Chest X-Ray and CT Scan Identification of COVID-19

**DOI:** 10.1155/2021/5528144

**Published:** 2021-06-04

**Authors:** Woan Ching Serena Low, Joon Huang Chuah, Clarence Augustine T. H. Tee, Shazia Anis, Muhammad Ali Shoaib, Amir Faisal, Azira Khalil, Khin Wee Lai

**Affiliations:** ^1^Department of Electrical Engineering, Faculty of Engineering, University of Malaya, 40603 Kuala Lumpur, Malaysia; ^2^Department of Biomedical Engineering, Faculty of Engineering, University of Malaya, 40603 Kuala Lumpur, Malaysia; ^3^Department of Biomedical Engineering, Faculty of Production and Industrial Technology, Institut Teknologi Sumatera, Lampung 35365, Indonesia; ^4^Faculty of Science and Technology, Universiti Sains Islam Malaysia, 71800 Nilai, Negeri Sembilan, Malaysia

## Abstract

Pneumonia is an infamous life-threatening lung bacterial or viral infection. The latest viral infection endangering the lives of many people worldwide is the severe acute respiratory syndrome coronavirus 2 (SARS-CoV-2), which causes COVID-19. This paper is aimed at detecting and differentiating viral pneumonia and COVID-19 disease using digital X-ray images. The current practices include tedious conventional processes that solely rely on the radiologist or medical consultant's technical expertise that are limited, time-consuming, inefficient, and outdated. The implementation is easily prone to human errors of being misdiagnosed. The development of deep learning and technology improvement allows medical scientists and researchers to venture into various neural networks and algorithms to develop applications, tools, and instruments that can further support medical radiologists. This paper presents an overview of deep learning techniques made in the chest radiography on COVID-19 and pneumonia cases.

## 1. Introduction

Pneumonia is life-threatening and one of the top diseases, which causes most deaths worldwide. It was projected that 1.4 million children die of pneumonia every year, in which 18% of the total children who died are below five years of age. In December 2019, at the epicentre in Wuhan, China, a novel coronavirus, severe acute respiratory syndrome–coronavirus-2 (SARS-CoV-2), causing COVID-19, emerged and is now a worldwide pandemic. As of 29^th^ September 2020, COVID-19 has been confirmed in 215 countries and territories, involving 33,558,131 cases with 1,006,471 deaths globally, which is a 3% mortality rate [1]. Most reported infections were in the USA, Brazil, India, Russia, South Africa, Mexico, Peru, Colombia, Chile, Spain, and many others [1]. Countries have declared emergencies and national lockdown while cases have been reported to increase at an alarming rate [2].

Pneumonia is the inflammation of the alveoli inside the lungs [3]. The inflammation will build up fluid and pus that subsequently causes breathing difficulties. The patient will show symptoms such as shortness of breath, cough, fever, chest pains, chills, or fatigue. Antibiotics and antiviral drugs can treat bacterial and viral pneumonia. COVID-19 was originally called novel coronavirus-infected pneumonia (NCIP) [3]. The symptoms are similar to other variations of viral pneumonia and more [4] of which include rapid heartbeat, breathlessness, rapid breathing—also known as acute respiratory distress syndrome (ARDS), dizziness, and heavy perspiration [3]. COVID-19 damages the cells and tissues that line the air sacs in the lungs [3]. The damaged cells and tissues can disintegrate and clot the lungs causing difficulties in breathing [3]. Nevertheless, an immediate diagnosis of COVID-19 and the consequent application of medication and treatment can significantly aid and prevent the deterioration of the patient's condition, which eventually can lead to death [5].

Hence, it is a challenge to diagnose a patient with COVID-19 via medical imaging. Deep learning models mimic human-level accuracy and precision in analysing and segmenting a medical image without human error [6]. However, deep learning cannot substitute medical professionals like physicians, clinicians, and radiologists in medical diagnosis [6], but it can assist medical experts in the field in executing and processing time-consuming works, such as determining chest radiographs for the signs of pneumonia and distinguishing the types of pneumonia and its severity [6].

## 2. Background of COVID-19

Coronaviruses are single-stranded ribonucleic acid (RNA) viruses, with the size of the virus approximately 26 to 32 kilobases. In late December 2019, a new (novel) coronavirus was identified in China, causing severe respiratory disease, including pneumonia. US Department of Health and Human Services/Centers for Disease Control and Prevention (CDC) reported that Chinese authorities declared an outbreak caused by a novel coronavirus, SARS-CoV-2 [7]. The coronavirus can cause mild to severe respiratory illness, known as Coronavirus Disease 2019 (COVID-19). The outbreak began in Wuhan, Hubei Province, China, and has spread to many countries worldwide—including Malaysia. World Health Organisation (WHO) declared COVID-19 a pandemic on 11 March 2020. CDC also stated the coronavirus could be spread mainly through close contact from person to person, face to face, and physically near each other within 6 feet [8].

The SARS-CoV-2 spreads more efficiently than influenza but not as efficiently as measles, one of the most contagious viruses. The respiratory ailment spreads throughout droplets of air. The infection is transmitted primarily via close contact and infects through respiratory droplets distributed in the air when a person coughs or sneezes. When a person contaminated with SARS-CoV-2 coughs, sneezes, sings, talks, or breathes, he or she produces respiratory droplets which range in size from large droplets visible to the human eye to smaller droplets. The tiny droplets can also form particles as they dry very quickly in the airstream [8]. Breathing difficulty is an indication of plausible pneumonia and requires prompt clinical deliberation and care. Research indicates that people suffering from COVID-19 often show hyperthermia and breathing problems [9]. Currently, there are no antibodies or definitive treatment for COVID-19 patients available to the public. The US Food and Drug Administration (FDA) had no authorised or approved vaccine to prevent COVID-19 [8] until 12 December 2020, when the Pfizer-BioNTech coronavirus vaccine, which offers up to 95% protection against COVID-19, has been authorised as safe, effective, and only for emergency use [10]. However, the World Health Organisation (WHO) encouraged the facilitation of vaccines by public persuasion instead of making the injections mandatory [11].

Early diagnosis of COVID-19 is critical to prevent human transmission of the virus to maintain a healthy population. Reverse transcription-polymerase chain reaction (RT-PCR) test is used to detect COVID-19 disease. It shows high specificity but is inconsistent with sensitivity in sensing the existence of the disease [12]. It demonstrates a certain proportion of false-negative results. However, when the pathological load is high during the symptomatic phase, the test is more accurate. The (RT-PCR) test kits are also limited in some geographical regions, especially third-world countries [13]. The turnaround time is 24 hours in major cities and is even longer in rural regions [9]. There is an urgency to explore other possibilities to distinguish the ailment and enable immediate referrals for the SARS-CoV-2-infected patient [9]. The chest X-ray plays a crucial role and is the first imaging technique to diagnose COVID-19 [14]. The virus presents on the Chest X-ray as ground-glass opacities, with peripheral, bilateral, and primary basal distribution [12]. These presentations seem comparable to those resulting from non-SARS-CoV-2-related viral, bacterial, fungal pneumonia [9, 12].

Furthermore, researchers found it problematic to differentiate viral pneumonia from other forms of bacterial and fungal pathogens [15]. Both chest X-ray and CT scan are not encouraged to be used as the primary diagnostic tool to screen/confirm and evaluate respiratory damage in COVID-19 because of the high risk and rapid increase in disease transmission [9, 13]. CT scans are discovered to be less explicit than RT-PCR but highly sensitive in sensing COVID-19 and can act as a fundamental role in disease analysis/treatment [13]. Nevertheless, the American College of Radiology has endorsed CT scans' practice as a primary-line assessment [16]. There are further concerns in using CT scans as a first-line test for the augmented risk of transmission, access, and cost, contributing to the recommendation [9]. As the pandemic became calamitous, radiological imaging is considered compulsory where portable chest X-rays are a useful and practical alternative [12]. However, the images' valuation placed a severe responsibility for radiological know-how, which is frequently lacking in regions with limited resources. Therefore, automated decision-making tools could be essential to appease some of this problem and to quantify and identify disease development [9].

### 2.1. Background on Deep Learning (DL)

Artificial intelligence (AI) is a computer science branch that allows machines to execute human intelligence tasks. With the evolution of AI and Internet-of-Things, medical equipment has rapidly changed, which provides many possibilities in medical radiology. Machine learning (ML) techniques can achieve the objective of AI. It is the subset of AI to allow computer systems with the learning ability and implement tasks with the data automatically without manual programming. Deep learning (DL) is a subset of machine learning related to methods simulating the neurons of the human brain [17, 18]. The implementation of ML is to apply DL as an essential subject with its technology in classification, recognition, and identification of images or videos. The algorithm instructs the information to process patterns impersonating the human neural system. DL is currently an essential subject with its technology in classification, recognition, and identification of images or videos. DL functions on algorithms for cognitive method simulation and data mining developing concepts [19]. DL maps input data consisting of hidden deep layers required to be labelled and analyzed concealed patterns within the complex data [20]. Between ML and DL, DL can automatically classify features and provide accurate results with high-end GPU help whereas ML requires a wider range of data to be preprocessed as the features need to be extracted manually. ML integrates various computational models and algorithms to mimic the human neural system whereas the DL-based network is more profound and is created with many hidden layers compared to conventional ANN. DL algorithms do not require many feature classifications and acquire directly from the data to display their higher problem-solving aptitudes. DL can interpret data and extract a wide range of dimensional features, notwithstanding if the features are visible or invisible to the naked human eye. This diminishes manual data preprocessing such as segmentation. DL can handle complex data representations and mimic trained physicians by identifying and detecting the features to make clinical decisions. DL architectures are applied in medical X-ray detection and various areas such as image processing and computer vision in medicine [17]. DL progresses in the medical sector to comprehend higher results, expand disease possibility, and execute valid real-time medical image [21, 22] in disease recognition systems [23].  Table 1 shows the neural network's significant contributions to deep learning [23, 24].

Figure 1 below shows the mind map of the types of machine learning and deep learning techniques created [25].

Convolutional neural network (CNN) most often apply to image processing problems where a computer identifies the object in an image. CNN can also be used in natural language processing projects as well. CNN modelling is adequate for processing and classifying images. A regular neural network has three layers: an input layer, a hidden layer, and an output layer. The input layer has different forms, whereas the hidden layer performs calculations on these inputs. The output layer delivers the outcome of the calculations and extractions. Each of the layers contains neurons and has its weight connected to the neurons in the previous layer. Hence, the data that is provided in the network does not produce assumptions via the output layer. However, the regular neural network cannot be applied if the data consists of images or languages. This is where convolutional neural network (CNN) comes in. CNN treats data as spatial data. Unlike regular neural network, the CNN neurons are not connected to every layer from the input layers to the hidden layers, and finally, the output layers only choose the neurons closest to it with the same weight. CNN upholds the spatial aspect of the dataset, which means that it undergoes a filtering process that simplifies complex images to better-processed images that are understood. The CNN is made up of many layers, consisting of several individual layers known as the convolutional layer, the pooling layer, and a fully connected layer. Inside, the layer of the CNN also consists of the rectified linear unit layer (ReLU). The ReLU layer activates the function to ensure nonlinearity as the data progresses through each layer in the network. Without ReLU, the data that is provided at the input layer would lose the dimensionality that is required in the network. The fully connected layer performs classification on the datasets. The CNN works by placing a filter over an array of image pixels and creating a convolved feature map. The analogy is like looking at an image through a window allowing specific features within the image to be seen. This is also known as the typical 2D convolutional neural network. The pooling layer reduces the sample size of the particular feature map, which speeds up the process by reducing the parameters the network needs. The output is the pool featured map, consisting of two execution methods, i.e., max pooling and average pooling. Max pooling takes the maximum input of a particular convolved feature, whereas the average pooling takes the convolved feature's average. The next step is feature extractions, whereby the network creates a picture of the image data based on its mathematical rules. The images' classification requires the network to move into the fully connected layer by flattening and simplifying the images. A complex set of neural network connections can only process linear data. If the data is unlabelled, unsupervised learning methods can be applied by using autoencoders to compile the data in a low dimension space performing calculations, then, additional layers are reconstructed to upsample the existing data.

CNN is the reason DL is so well known, but it has limitations and fundamental drawbacks. The max-pooling or successive convolutional layers lose valuable information. CNN needs a large amount of data to work, and it loses information in the pooling area, which in turn reduces spatial resolution, resulting their outputs to be invariant to small changes in the inputs. Currently, the issue is addressed by building complex architectures around CNNs to recover the lost information.

Generative adversarial network (GAN) trains two networks which comprise the artificial data samples that resemble data in the training set and the discriminative network that distinguishes the artificial and the original model: in simple means, GAN has a generator data, and the other is the discriminative data. The generator data is the counterfeiter that consistently produces artificial data, and the discriminator will try to expose the counterfeiter. Each time the discriminator manages to identify the image as a counterfeit, the generator will keep improving it until it is as accurate as possible.

Capsule networks is an artificial neural network that is significantly new. It is a network that applies local capsules in an artificial neural network that consists of complicated internal computations on the inputs and encapsulates these computations' results into a small vector of highly informative outputs. CapsNet architecture reached state-of-the-art performance on MNIST and had better performance than CNNs on MultiMNIST [26].

## 3. Radiology Perspective of Coronavirus Disease 2019 (COVID-19)

In December 2019, a lower respiratory tract feverish illness of unfamiliar derivation was informed in a cluster of patients in Wuhan City, Hubei Province, China. Coronavirus disease 2019 (COVID-19) is accountable for this epidemic to date. Other corresponding pulmonic conditions have been documented as being triggered by other strains of the coronavirus family. The most notable instances are the severe acute respiratory syndrome (SARS) and the Middle East respiratory syndrome (MERS). The SARS epidemic was under control with no human contaminations reported since 2003 whereas minor MERS occurrences continue to be stated. Hence, imaging is an essential analytical procedure tool observing disease development and coronavirus-related pulmonary syndrome [27]. Imaging structures in critical and chronic phases of SARS and MERS are inconsistent and inexplicit [28]. The first accounts of imaging discoveries of COVID-19 have also been described as inconclusive [29–31]. Researchers are conducting various studies to distinguish further and identify the imaging features of this new coronavirus syndrome, but the information is still inadequate.

The incident of COVID-19 intensified beyond human beings comprehension; more clusters and incidences are reported daily by the several ten thousand in some parts of the world. The disorder's etiologic and medical structures are comparable to SARS and MERS; the knowledge and aptitude from those pulmonary syndromes can support handling the sharp increase of COVID-19 eruption. This review segment will allow us to be familiar with the radiologist and imaging spectrum of coronavirus syndromes and discuss the reported imaging features of COVID-19.

SARS was discovered in 2003 as the first epidemic of the new era in Guangdong Province, China, which its clinical discovery presented as novel viral pneumonia. The clinical disease-infested 8,422 individuals demanded 916 lives before it was confined, and no occurrence has been reported ever since [32]. MERS was revealed in Saudi Arabia, where a patient's sputum consisted of the novel coronavirus in 2012 [32]. The disease has infected 2,492 individuals worldwide, and 858 human lives were lost, as the latest discovery was reported in December 2019 [32].

There are various imaging features of SARS and MERS that share similarity to one another, but some differences are shown in Table 2. The analysis of COVID-19 is hypothesised on the foundation of indications of pneumonia (e.g., dry cough, lethargy, myalgia, malaise, and dyspnea similar to symptoms of SARS and MERS) as well as past travelling activities to China or acquaintance with a COVID-19 patient. The development of the diseases and their severity rely on chest imaging to acquire valuation, discovery, and identification. A portable chest X-ray (CXR) is used as the first-line modality for COVID-19 patients instead of CT scans, as CT scans are applied in specific situations. Portable chest X-ray (CXR) has the benefit of discarding patients' need to travel from one location to another and diminish the use of personal protective equipment (PPE). The arrangement is to avoid nonessential imaging and transportations to the radiology department. Czawlytco et al. discovered that chest X-ray is insensitive in the early detection of COVID-19 with a sensitivity of only 59% [33]. Chest X-ray is not recommended for patients with flu/influenza-like symptoms. It is also not recommended to be used on confirmed COVID-19 patients with mild symptoms. Therefore, chest X-ray is designated for COVID-19 patients with acute respiratory status or COVID-19 patients with mild symptoms but has high-risk factors for developing severe disease. Chest radiography and tomography cannot be used as first-line screening or diagnosis in COVID-19, even with a normal chest X-ray and CT images, the possibility of COVID-19 cannot be ruled out as a patient might be asymptomatic, and the lung condition maintains to be expected. However, information of COVID-19 patients initially declared hostile on the virus using the real-time reverse transcriptase-polymerase chain reaction (RT-PCR) was discovered to have COVID-19 via early CT findings [32]. In the meantime, initial findings in imaging may show normal conditions of the lungs. Hence, standard chest imaging does not rule out the possibility of being infected with SARS-CoV-2 [32].

### 3.1. Artificial Intelligence on Chest X-Ray (CXR) and CT Scans

With the struggle against the SARS-CoV-2 rapid infection, active screening and immediate medical response for the infected patients are desperately needed. RT-PCR is a common screening application which is manual, time-consuming, intricate, and arduous with only a 63% positivity rate [34, 35]. Research regarding early identification of COVID-19 by using CXR and other imaging modalities is still in development. The Guardian reported information shared by a respiratory physician that SARS-CoV-2 pneumonia is different from common viral pneumonia cases [36]. However, the images of several viral cases of pneumonia are comparable with other infectious and inflammatory lung diseases [34]. The COVID-19 symptoms being similar to other viral pneumonia can result in wrong diagnosis and prognosis in many hospitals, especially in the emergency department which is overloaded and understaff [34].

Today, many biomedical problems and complications such as brain tumour detection, lung disease detection, breast cancer detection, and other oncological emergencies are using artificial intelligence (AI) solutions [34]. Convolutional neural network (CNN), a deep learning technique, has been advantageous in revealing image features that are not obvious in the original image [34]. The accuracy of the deep learning algorithm relies on imaging quality, and CNN can improve imaging quality in low-light images from a high-speed video endoscopy, discover pulmonary nodules through CT images, identify paediatric pneumonia from CXR images, and automatically labelling of polyps in a colonoscopy and cystoscopic image analysis from videos [34]. Hence, only confirmed positive COVID-19 patients' images were selected. Wang et al. (2017) have shown to accumulate datasets that allow significant developments in medical imaging tools to progress in the prediction of various pneumonia and the outcome towards the infected patient [37, 38]. Rajpurkar et al. (2017) and Cohen et al. (2019) works on both organised models to foresee various pneumonia [37, 39, 40]. Deep learning models and algorithms are tools that can be developed for triage cases during the shortage of physical tests, particularly RT-PCR [37, 41, 42]. The American College Radiology (ACR) only recommended portable CXR in an ambulant care facility when required and strongly discourage CT to apply and inform decisions on a suspected COVID-19 patient and whether or not to conduct RT-PCR test, admit the patient, provide other treatment, and dissuade the patient from being quarantines or others [33]. However, deep learning models and algorithms should predict patient outcomes and permitting the physician to immediately facilitate care and management [37, 43]. COVID-19 can be considered in extraordinary extreme situations, where physicians could be faced with decisions to select which patient to assign for which healthcare resources based on the severity level [43]. The tools would serve to monitor the development of SARS-CoV-2 positive patients' ailment evolution [37].

### 3.2. Approached Techniques and Convolutional Neural Network Architecture

Deep learning (DL) is a subsection of machine learning, and a convolutional neural network is a type of deep learning commonly applied in the computer vision domain. Examples of CNN architectures are LeNet, AlexNet, GoogLeNet, Visual Geometry Group (VGG) Net, ResNet, and others [44]. The goal is to apply deep learning neural network architectures to create practical applications to improve diagnosis and prognosis performance [44].

Deep CNN was created with LeNet designed to recognise handwritten digits. However, LeNet has limitations, and thus, its successor AlexNet was the first deep CNN that accomplished outstanding results for the organisation and recognition tasks on the image. Due to hardware limitations in early 2000, deep CNN architectures' learning capacity was restricted to small sample size images. AlexNet was made applicable to all types of images—its depth was extended from LeNet's five layers to eight layers: five convolutional layers, two fully connected hidden layers, and one fully connected output layer generalised for different image resolutions. However, it caused overfitting issues. The overfitting issue was fixed with the dropout algorithm, which arbitrarily eliminated some transformational units during the training process. DenseNet is a modern CNN architecture that requires fewer visual object recognition parameters. It is the product of the previous layer that combines with the output of a future layer. The objective of DenseNet is to recognise visual objects by densely connecting all the layers. ResNet is known as the residual net, which divides a layer into two branches, where one branch does nothing to the signal, and the other processes ResNet adds the previous layer with the future layers. Usually, a deep neural network tends to randomly overfit and sometimes produce more preliminary results than a network with a few layers.

CNN is based on biological processes of the visual cortex of the human and the animal brain. CNN consists of multiple layers where a higher layer is connected to a lower layer to study abstract features of the images by considering the spatial relationships between the receptive fields. This allows CNN to recognise patterns and identify images within the layers of images. Various CNN models apply different layers, number of neurons, and receptive fields in the respective layers and algorithm [44]. Integrating transfer learning into the technique modifies the CNN models applied to pretrain many radiology image datasets to diagnose COVID-19 problems [44]. This technique bypasses the hassle to train all the images from scratch everytime new cases or images are identified. However, this method is not valid with the amount of radiology images dataset available for the public.

Based on the studies in Table 3, several studies use deep learning for COVID-19 diagnosis using radiology images.

Table 3 includes some research conducted with deep learning models using two types of medical images, i.e., chest-X-ray (CXR) and CT images. Based on the table, the majority of the researchers used CXR images because of their availability. The CXR requires low memory space and high results performance which reassure researchers to apply these images into the respective deep learning models. There are a total of 52 researches using various deep learning methods to achieve results. Out of the 52 journals mentioned above, 34 of the studies used CXR images, 17 studies used CT images, and 4 of the studies used CT and CXR images. More CXR images from COVID-19 patients found in the public databases encouraged researchers to study deep learning utilising these images. Journals from the medical field often mentioned that CT images show higher accuracy performance, but these accuracies were debunked because it was not explicitly shown in the deep learning-based CAD systems. The nature of the CT images that produce many cross-sections just for one patient result in high memory usage for the facility to handle. In general, CT images were previously deemed more accurate than CXR images because the CT images' cross-section images are individually labelled. Hence, studies that utilised the combination of CT and CXR images show promising results. However, studies with 3D data have lower performance than 2D data, mainly because there are primarily 2D data available for the public to use. The table also shows that deep learning models produced more stable results with more data.

### 3.3. COVID-19 Radiology Data Sources for Potential Modelling

This section describes the radiology imaging data source available for researchers to exploit the capabilities of deep learning techniques using CNN architectures to overcome COVID-19. The variability of the data requires different AI methods to study. Radiology images like CXR and CT images are high-dimensional data requiring CNN-based models to process the images like LeNet, AlexNet, GoogLeNet, VGGNet, and ResNet [44]. AlexNet is a category of CNN designed by Alex Krizhevsky in 2012. It is a popular CNN that sets the essential milestones to its incomers like network-in network [89] by Lin et al. [90], VGGNet [91] by Simonyan et al., and GoogLeNet (Inception v-1) by Szegedy et al.

CNN architecture application requires a large dataset for training, testing, and validating.  Table 4 describes the available data sources for COVID-19 radiology images, mainly CXR and CT images.

The data sources depicted in Table 4 are the standard open-source radiology images available for the public to access, study, and characterise using CNN architectures. However, based on the table, there are minimal COVID-19 data to comprehensively utilise AI techniques to conduct an intensive study. This creates concerns and difficulties when utilising these techniques in real-world practice with a limited number of datasets available.

## 4. Challenges in the Interpretation and Application of Imaging Features of COVID-19 and Suggestions to Overcome

In theory, utilising AI is to eliminate fake news that can be found on the worldwide web and various social media platforms to ensure authenticity, responsible, and dependable information about the pandemic. However, scientists face many challenges and limitations shown in Table 5 below to produce ethical and reliable results for the public.

When implementing a DL model, test and train images from the same goal are used to distribute data and predict the medical images into their respective categories. The idea is impossible to achieve due to limited data availability or weak labels [9]. Despite many cases happening worldwide, we have very limited COVID-19 CXR or CT image data publicly available. Therefore, it is difficult to train the DL models and distinguish the images between COVID-19-related CXR and CT and non-SARS-CoV-2 viral, bacterial, and other pathogen-related CXR and CT images. The Radiological Society of North America (RSNA) [97] and Imaging COVID-19 AI Initiative in Europe [98] are aimed at providing easily accessible data to the public. These data allow various features across categories to enhance interclass variance, leading to better DL performance. Due to lack of data, the model will overfit and produce weakly generalised results [99]. Hence, data augmentation has been proven to be effective in training discriminative DL models. Examples of data augmentation techniques are flipping, rotating, colour jittering, random cropping, elastic distortions, and generative adversarial network- (GAN-) based synthetic data generation [100]. Medical images found in ImageNet have different visual characteristics showing high interclass similarities [101]. Thus, traditional augmentation methods that perform simple image alterations are less effective [102]. GAN refers to the specialised algorithms and cavernous learning systems towards the compelling predictions and transformation of data from one to another that produce dynamic data and images so that better recognition and analysis can be done. GAN-based DL models are applied to generate data artificially. Therefore, to overcome the data-scarce situation, GAN is used to develop effective data augmentation strategies for medical visual recognition.

Based on the journal written by Afshar et al., CNNs that were applied to identify positive COVID-19 CXR images are prone to lose spatial information between image instances and require a large dataset to compensate for the loss. Capsule networks, a.k.a COVID-CAPS, is an alternative modelling framework capable of handling small datasets. Capsule network consists of capsules in the convolutional layers. It has the potential to improve further diagnosis capabilities. Hence, using capsule network to pretrain the images is expected to improve the accuracy where each capsule in the convolutional layers represents a specific image instance at a specific location through several neurons. The routing agreement in the capsule network helps CNN models to identify spatial relations.

## 5. Conclusion and Future Works

COVID-19 has disrupted the lives of people worldwide. The number of casualties related to the disease cannot be contained and has increased by the thousands daily. AI technologies have existed to help us live comfortably and have many successes and contributions in streamlining processes and procedures. However, the spread of COVID-19 is exceptionally lethal as it transmits faster and broader than ever. The coronavirus is also continuously revolutionising with new spikes, and protein mutations have been reported in countries like Malaysia, United Kingdom, South America, Australia, the Netherlands, and Singapore. The clinical impact of this discovery and its infectivity or aggressiveness is still unknown. Whether or not the mutation will affect the development of radiography imaging is also still a mystery.

Based on the worldmeter website: https://www.worldometers.info/coronavirus/, some countries failed to respond to the disease, some are barely tackling the situation, and some are handling the situation much more successfully. Hence, a country that managed to have the situation under control might experience a spike increase overnight if society became lenient in taking proper measures.

Although many researchers have published their works, the number of contributions and AI applications towards tackling COVID-19 is rudimentary. With the petrifying number of deaths and infected patients discovered daily and the virus's mutation undergoing speedily and unknowingly, we are nowhere near applying AI on radiography imaging to identify that the patient is infected with SARS-CoV-2. The development of AI and radiography imaging is slow due to the limited availability of COVID-19 datasets. With the number of people affected worldwide, AI methods require massive data and several computational models and CNN architectures to learn and acquire knowledge. The current data that most researchers acquired from open-source websites is insufficient. Even with the best available data, it is far from perfect; as the data alone cannot explain the pandemic's whole situation. Therefore, for future research and development, in terms of acquiring radiography imaging data, the best way is to have access to reliable, global, open data, and research to build an infrastructure that allows researchers who are experts in the field of radiology, artificial intelligence, deep learning, and imaging to navigate and understand this data and its development.

Most of the COVID-19 radiography image datasets are stored in different formats, standards, sizes, and quality, which are obstacles for scientists to speed up development for COVID-19-related AI research. Therefore, in future development, COVID-19 radiography images should have standard operating procedures to allow researchers or scientists and anyone who has the passion and are interested to contribute and utilise the information freely. A future study on deep learning models identifying and distinguishing the difference between COVID-19 images and viral pneumonia is essential. The study would help radiologists and physicians understand the virus and evaluate future coronaviruses using CT and CXR images more efficiently and effectively.

## Figures and Tables

**Figure 1:** Mindmap of machine learning (ML) algorithm created by Robert Herman from mind meister [25].

**Table 1:** Significant contributions of the neural network to deep learning [23, 24].

Milestone/contribution	Year
McCulloch-Pitts neuron	1943
Perceptron	1958
Backpropagation	1974
Neocognition	1980
Boltzmann machine	1985
Restricted Boltzmann machine	1986
Recurrent neural networks	1986
Autoencoders	1987
LeNet	1990
LSTM	1997
Deep belief networks	2006
Deep Boltzmann machine	2009

**Table 2:** Comparison of clinical and radiological features of COVID-19, SARS, and MERS [32].

Feature	COVID-19	SARS	MERS
Clinical sign or symptom			
Fever or chills	Yes	Yes	Yes
Dyspnea	Yes	Yes	Yes
Malaise	Yes	Yes	Yes
Myalgia	Yes	Yes	Yes
Headache	Yes	Yes	Yes
Cough	Dry	Dry	Dry or productive
Diarrhoea	Uncommon	Yes	Yes
Nausea or vomiting	Uncommon	Yes	Yes
Sore throat	Uncommon	Yes	Yes
Arthralgia		Yes	Uncommon
Imaging finding			
Acute phase			
Initial imaging			
Normal	15–20% of patients	15–20% of patients	17% of patients
Abnormalities			
Common	Peripheral multifocal airspace opacities (GGO, consolidation, or both) on chest radiography and CT.	Peripheral multifocal airspace opacities (GGO, consolidation, or both) on chest radiography and CT.	Peripheral multifocal airspace opacities (GGO, consolidation, or both) on chest radiography and CT.
Rare	Pneumothorax	Pneumothorax	Pneumothorax
Not seen	Cavitation or lymphadenopathy	Cavitation or lymphadenopathy	Cavitation or lymphadenopathy
Appearance	Bilateral, multifocal, basal airspace; normal chest radiography findings (15%)	Bilateral, multifocal basal airspace on chest radiography or CT (80%); isolated unilateral (20%)	Unilateral, focal (50%); multifocal (40%); diffuse (10%)
Follow-up imaging appearance	Persistent or progressive airspace opacities	Unilateral, focal (25%); progressive (most common, can be unilateral and multifocal or bilateral with multifocal consolidation)	Extension into upper lobes or perihilar areas, pleural effusion (33%), interlobular septal thickening (26%)
Indications of poor prognosis	Consolidation (vs. GGO)	Bilateral (like ARDS), for or more lung zones, progressive involvement after 12 d	Greater involvement of the lungs, pleural effusion, pneumothorax
Chronic phase	Unknown, but pleural effusion and interlobar septal thickening have not yet been reported		
Transient reticular opacities		Yes	Yes
Air trapping		Common (usually persistent)	
Fibrosis	More than one-third of patients	Rare	One-third of patients

Note: SARS: severe acute respiratory syndrome; MERS: Middle East respiratory syndrome; COVID-19: coronavirus disease 2019; GGO: ground-glass opacity; ARDS: acute respiratory distress syndrome [32].

**Table 3:** Summary of deep learning methods and CNN architectures for COVID-19 using radiology images. CT images are computer tomography images, and CXR images are chest X-ray images.

No.	Papers	Data	Types of images	AI methods to establish the algorithm	CNN architecture	Results for detecting COVID
1	[44, 45]	Total images: 4,356, COVID-19 images: 1,296, pneumonia images: 1,735, nonpneumonia images: 1,325	CT	3D deep learning	ResNet-50 and COVNet	Area under the curve (AUC): 0.96

2	[44, 46]	Total images: 618, COVID-19 images: 219, influenza-A (H1N1, H3N2, H5N1, H7N9, and others), images: 224, normal healthy lungs images: 175	CT	3D CNN model for segmentation	Location-attention network and ResNet-18	Accuracy of 86.7%, average time: 30 s

3	[44, 47]	(PA) posterior-anterior images: 5,941, normal images: 1,583, bacterial pneumonia images: 2,786, non-COVID-19 viral pneumonia images: 1,804, COVID-19 images: 68	CXR	Drop weights based Bayesian CNNs	Bayesian ResNet50V2	Accuracy of 89.92%

4	[44, 48]	COVID-19 images: 453, training images: 217	CT	Inception migration-learning model		Internal validation: accuracy: 82.9%, specificity: 80.5%, sensitivity: 84%; External testing dataset: accuracy: 73.1%, specificity: 67%, sensitivity: 74%

5	[44, 48]	Total images: 1,065, COVID-19 images: 325; viral pneumonia images: 740	CT	Modified inception transfer-learning model		Accuracy: 79.30%, specificity: 0.83, sensitive: 0.67

6	[44, 49]	Total patients: 133, severe/critical patients: 54, nonsevere/critical patients: 79	CT	Multilayer perception and long short term memory (LSTM)		Area under the curve (AUC): 0.954

7	[44, 50]	Total images: 4,266, COVID-19 images: 2,529, CAP images: 1,338, influenza A/B images: 135, standard images: 258, total patients: 3,177, COVID-19 patients: 1,502, influenza A/B patients: 83, CAP patients: 1,334, healthy subjects: 258	CT	2D deep learning CNN	ResNet 152	Accuracy: 94.98%, AUC 97.71%, sensitivity: 90.19%, specificity: 95.76%, the average time is taken to read: 2.73 s

8	[44, 51]	Total 1,136 cases from 5 hospitals, COVID-19 images: 723, non-COVID-19 images: 413	CT	3D deep learning method	UNet ++ & ResNet-50	Specificity: 0.922, sensitive: 0.974

9	[44, 52] ,	COVID-19 patients: 50, ordinary people: 50,	CXR	5 pretrained CNN	ResNet-50, ResNet101, ResNet52, InceptionV3, and inception-ResNetV2	ResNet-50: accuracy: 98.0%
10	[44, 53]	Total images:13,975, total patients:13,870	CXR	Deep learning CNN	COVID-net	Accuracy: 92.4%

11	[44, 54]	Total patients: 157	CT	CNN	ResNet-50	Area under the curve (AUC): 0.996

12	[34, 44]	Normal images: 1,341, viral pneumonia images: 1,345, COVID-19 images: 190	CXR	CNN	AlexNet, ResNet-18, DenseNet-201, SqueezeNet	Accuracy: 98.3%

13	[44, 55]	Total COVID-19 images: 531, CXR images: 170, CT images: 361	CT and CXR	CNN with transfer learning	Pretrained AlexNet	Accuracy: CXR images: 98.3%, CT image: 94.1%

14	[6]	Total images: 5,232, normal images: 1,346, bacterial pneumonia images: 2,538, viral pneumonia images: 1,345	CXR	Deep learning framework using transfer learning	Pretrained on ImageNet, trained using AlexNet, ResNet18, inception V3, DenseNet121, GoogLeNet, and ensemble model	Ensemble model: accuracy: 96.4%, recall: 99.62% (unseen data)

15	[5]	Total images: 5,247, bacterial pneumonia images: 2,561, viral pneumonia images 1,345, normal images: 1,341	CXR	Pretrained deep CNN and used for transfer learning	AlexNet, ResNet18, DenseNet201, and SqueezeNet	DenseNet201 accuracy: normal and pneumonia: 98%, normal images, bacterial, and viral pneumonia: 93.3%, bacterial and viral pneumonia: 95%

16	[17]	Total images: 306, COVID-19 images: 69, normal images: 79, bacterial pneumonia images: 79, viral pneumonia images: 79. The dataset number increases to 8,100 images after using the GAN network.	CXR	Deep transfer learning: using GAN network to generate more images to help detect the virus. Three deep transfer models.	AlexNet, GoogLeNet, Restnet18 with performance measures in different scenario and classes	GoogLeNet accuracy: 80.56%

17	[56]	Dataset was collected from medRix and bioRxiv; COVID-19 images: 349, total patients: 216	CT	Multitask learning and self-supervised	DenseNet-169, ResNet-50	F1 score: 0.90, AUC: 0.98, accuracy: 0.89

18	[36]	Total images: 2,200, COVID-19 images: 800, viral pneumonia images: 600	CT	Machine learning technique using Microsoft Azure	ResNet	High accuracy: 91%, overall accuracy: 87.6%

19	[57]	Total images: 15,495, normal images: 12,544, COVID-19 image: 2,951	CXR	CNN model	UNet, UNet++, DLA, DenseNet-121, CheXNet; inception-v3, ResNet-50	F1 score: 85.81%, sensitivity: 98.37%, specificity: 99.16%

20	[58]	Diverse datasets from a different source	CT	Deep fully convolutional networks (FCN)	UNet, ResDense FCN	DSC: 0.780, sensitivity: 0.822, specificity: 0.951

21	[59]	Total images: 954, COVID-19 images: 308, normal images: 323, pneumonia images: 323 images	CXR	Deep learning modules using stacked architecture concept	DenseNet; GoogleNet	Sensitivity: 0.91, specificity: 0.95, F1 score: 0.91, AUC: 0.97
22	[52]	Total images: 7,406, COVID-19 images: 341, normal images: 2,800, viral pneumonia images: 1,493, bacterial pneumonia images: 2,772	CXR	2D five pretrained CNN based models	ResNet50, ResNet101, ResNet152, InceptionV3, and inception-ResNetV2	COVID-19 and normal: accuracy: 96.1%, COVID-19 and pneumonia accuracy: 99.5%, COVID-19 and bacterial accuracy: 99.7%

23	[60]	Total images (COVID-19, pneumonia, and normal): 1,266, COVID-19 images: 924	CT	3D pretrained the deep learning system and validate it.	DNN	Sensitivity (train): 78.93%, specificity (train): 89.93%, sensitivity (val): 80.39%, specificity (val): 81.16%

24	[61]	Total images (COVID-19, bacterial, and normal): 275, COVID-19 images: 88	CT	2D pretrained ResNet 50 using the feature pyramid network (FPN)	DRE-net	Sensitivity: 93%, specificity: 96%, accuracy: 99%

25	[62]	Total images: 624, COVID-19 images: 50	CXR	2D GAN + TL	AlexNet, GoogLeNet, ResNet18, SqueezeNet	Accuracy: 99%

26	[63]	Total images (COVID-19, bacterial, and normal): 1,427, COVID-19 images: 224, bacterial and viral pneumonia images: 714	CXR	2D transfer learning (TL)	VGG19, MobileNet, Inception, Xception, Inception ResNet v2.	Sensitivity: 98.66%, specificity: 96.46%, accuracy: 94.72%

27	[64]	Total images (COVID-19, pneumonia, normal): 6,008, COVID-19 images: 184	CXR	2D transfer learning (TL)	Three ResNet models	Accuracy: 93.9%

28	[65]	Total images (COVID-19, pneumonia, and normal): 8,850, COVID-19 images: 498	CXR	2D convolutional autoencoder (CAE)	AE: COVIDomaly	Accuracy: 76.52%

29	[66]	Total images (COVID-19, pneumonia, and normal): 2,905, COVID-19 images: 219	CXR	2D	CNN + k-NN + SVM	Accuracy: 98.70%

30	[67]	Total images (COVID-19, pneumonia, and normal): 2,905, COVID-19 images: 219	CXR	2D using hyperparameters Bayesian optimisation algorithm	ANN + AlexNet	Sensitivity: 89.39%, specificity: 99.75%, accuracy: 98.97%, F-score: 96.72%

31	[68]	Total images (COVID-19, pneumonia, and normal): 502, COVID-19 images: 180	CXR	2D patch-based convolutional neural network	ResNet-18	Sensitivity: 76.90%, specificity: 100.00%

32	[69]	Total images (COVID-19, pneumonia, and normal): 2,905, COVID-19 images: 219	CXR	2D	Ensemble: Resnet50 and VGG16	Sensitivity: 91.24%, specificity: 99.82%

33	[70]	Total images (COVID-19 and normal): 2,492, COVID-19 images: 1,262	CT	2D	TL and DenseNet201	Accuracy: 99.82%

34	[71]	COVID-19, pneumonia, and normal images from Cohen et al. [37]	CXR	2D	Xception	Sensitivity: 97.09%, specificity: 97.29%, accuracy: 97.40%
35	[72]	Total images (COVID-19 and normal): 380, COVID-19: 180	CXR	2D	5 pretrained models+ SVM	Accuracy: 94.7%

36	[73]	Total images (COVID-19, pneumonia, normal, and non-COVID-19): 2,905, COVID-19 images: 219	CXR	2D pretrained models such as ResNet101, Xception, InceptionV3, MobileNet, and NASNet	InstaCovNet-19	Accuracy: 99.08%, accuracy: 99.53%

37	[74]	Datasets contain COVID-19, pneumonia and normal images.	CXR	2D	5 pretrained CNNs	Accuracy: 95.00%

38	[75]	Datasets contain bacterial pneumonia, non-COVID viral pneumonia, and COVID-19 images.	CXR	2D	5 COVID-CAPS	Sensitivity: 90%, specificity: 95.8%, accuracy: 95.7%

39	[76]	Total images (COVID-19 and normal): 5,000, COVID-19 images: 184	CXR	2D	5 TL + pretrained models	Sensitivity: 100%, specificity: 98.38%

40	[55]	Total images (COVID-19 and normal): 526, COVID-19 images: 238	CXR + CT	2D	TL + AlexNet model	Sensitivity: 72%, specificity: 100%, accuracy: 94.1%

41	[77]	Total images (COVID-19 and normal): 320, COVID-19 images: 160	CXR + CT	2D Apache spark framework	TL + inceptionV3 & ResNet5	Sensitivity: 72%, specificity: 100%, accuracy: 99.01%

42	[78]	Total images (COVID-19, pneumonia, and normal): 4,575, COVID-19 images: 1,525	CXR	2D CNN used for deep feature extraction, and LSTM is used for detection using the extracted feature	LSTM+CNN	Sensitivity: 99.2%, specificity: 99.9%, accuracy: 99.4%

43	[79]	Dataset 1 images (COVID-19, pneumonia, and normal): 4,448, COVID-19 images: 2,479, dataset 2 images (COVID-19, pneumonia, and normal): 101, COVID-19 images: 52	CXR	2D	3D inception V1	Dataset 1: accuracy: 99.4%; dataset 2: sensitivity: 98.08%, specificity: 91.30%, accuracy: 93.3%

44	[80]	Total images (COVID-19, pneumonia, and normal): 1,343, COVID-19 images: 446	CXR	2D	Conditional GAN: LightCovidNet	Accuracy: 97.28%

45	[81]	Total images (COVID-19 and normal): 8,504, COVID-19 images: 445	CXR	2D	TL VGG-16 model	Sensitivity: 98.0%, specificity: 100.00%, accuracy: 94.5%

46	[82]	Total images (COVID-19 and normal): 746, COVID-19 images: 349	CT	2D	TL+ ensemble of 15 pretrained models: EfficientNets(B0-B5), NasNetLarge, NasNetMobile, InceptionV3, ResNet-50, SeResnet 50, Xception, DenseNet121, ResNext50, and Inception_resnet_v2	Accuracy: 85.0%
47	[83]	Total images (COVID-19 and normal): 2,482, COVID-19 images: 1,252	CT	2D	AE + random forest	Specificity: 98.77%, accuracy: 97.87%

48	[84]	Total images (COVID-19 and normal1): 50, COVID-19 images: 25	CXR	3D	COVIDX-net	Sensitivity: 100.00%, specificity: 80.00%

49	[85]	Total images (COVID-19 and Normal): 800, COVID-19 images: 400	CXR	2D using modern and traditional machine learning methods: (ANN), (SVM), linear kernel and (RBF), *k*-nearest neighbor (*k*-NN), decision tree (DT), and CN 2 rule inducer techniques	Deep learning models: MobileNets V2, ResNet50, GoogleNet, DarkNet, and Xception	ResNet50 accuracy: 98.8%

50	[86]	Total images (COVID-19 and Normal): 800, COVID-19 images: 400	CXR	2D CLAHE and Butterworth bandpass filter was applied to enhance the contrast and eliminate the noise.	The hybrid multimodal deep learning system COVID-deep net system.	Sensitivity: 99.9%, specificity: 100.0%, accuracy: 99.3%

51	[87]	Datasets from Cohen et al. [37]. Total images (COVID-19 and normal): 800, COVID-19 images: 400	CXR	2D benchmarking and diagnostic models: decision matrix that embedded a mix of 10 evaluation criteria and 12 diagnostic models, also known as multicriteria decision making (MCDM)	TOPSIS is applied for benchmarking and ranking purpose, while entropy is used to calculate the criteria's weights. SVM is selected as the best diagnosis model	Coefficient value: 0.9899

52	[88]	Total images (COVID-19 and normal): 800, COVID-19 images: 400	CXR	2D hybrid deep learning framework, pretrained deep learning models incorporating of a ResNet34, and high-resolution network model	COVID-CheXNet system	Sensitivity: 99.98%, specificity: 100.0%, accuracy: 99.99%

**Table 4:** Available data sources about COVID-19 radiology images for both chest X-ray and CT images.

No.	Sources	Data type	No. of images	Image type	Types of images	Links
1	J. P. Cohen's GitHub	Viral pneumonia (SARS, varicella, influenza) and COVID-19, bacterial pneumonia (Streptococcus spp., Klebsiella spp., Escherichia coli, Mycoplasma spp., Legionella spp., unknown, Chlamydophilla spp.) and COVID-19, fungal (Pneumocystis spp., lipoid) and COVID-19	Raw images: 910, annotated images: 210	jpg and png	CXR	https://github.com/ieee8023/covid-chestxray-dataset

2	European Society of Radiology	Total cases or images unknown	N/A	pdf	CXR and CT	https://www.eurorad.org/advanced-search?search=COVID

4	Kaggle	Posterior-anterior (PA), anterior-posterior (AP) lateral for X-rays and axial or coronal for CT scans	Normal images: 1,576, pneumonia ARDS images: 2, viral pneumonia images: 1,493, COVID-19 images: 58, SARS images: 4, bacterial pneumonia images: 2,772, bacterial Streptococcus images: 5	png, jpg, jpeg, and others	CXR and CT	https://www.kaggle.com/bachrr/covid-chest-xray

5	UCSD-AI4H	Total: 349 images from 216 patients	COVID-19 images: 349, non-COVID-19 images: 397	jpg and png	CT	https://github.com/UCSD-AI4H/COVID-CT

6	MedSeg	Images were segmented by a radiologist using 3 labels: ground-glass (mask value = 1), consolidation (=2), and pleural effusion (=3).	Image volumes—9 volumes, a total of >800 slices, COVID-19 masks 350 annotated slices. Lung masks > 700 annotated slices	jpg	CT	http://medicalsegmentation.com/covid19/

7	COVID-19 Radiography Database		COVID-19 images: 219, normal images: 1,341, viral pneumonia images: 1,345	png	CXR	https://www.kaggle.com/tawsifurrahman/covid19-radiographydatabase

**Table 5:** Challenges of radiology imaging addresses and AI applications.

No	Applications	Type of data	Challenges	AI methods	Sources
1	COVID-19 early detection using radiology images. Typically CXR and CT images	CXR images	Limited availability of annotated medical images and medical image classification remains the biggest challenge in medical diagnosis.	DeTraC deep convolution neural network	[14]
2		CXR images	Finding optimal parameters for the SVM classifier can be seen as a challenge. Finding optimal parameters for the SVM classifier can be seen as a challenge. Finding optimal values for the relief algorithm can be seen as another limitation of the study	COVIDetectioNet	[92]
3		CT images	Redundant data such as interferential vessels can be misdiagnosed as pathology. Radiologists have difficulty differentiating COVID-19 and other atypical and viral pneumonia diseases, which are the same in CT imagery and have similar symptoms.	AlexNet, VGG-16, VGG-19, SqueezeNet, GoogleNet, MobileNet-V2, ResNet-18, ResNet-50, ResNet-101, Xception	[93]
4		CXR images	Due to the sudden existence and infectious nature of COVID-19, systematic collection of the extensive data set for CNN training is formidable. Biomarkers found in the CXR images can be misleading.	Patch-based convolutional network	[68]
5		CXR images	The research is dealing with images taken directly from patients with severe COVID-19 or some form of pneumonia. However, in the real world, more people are unaffected by pneumonia. The limited number of data available provides a limitation to provide feasible results.	Multiclass classification and hierarchical classification, using texture descriptors and also pretrained CNN model	[94]
6		CXR images	Insufficient pulmonary diseases data limit us to conduct verification techniques.	Localise the areas in CXR symptomatic of the COVID-19 presence	[95]
7		CT images	Shortage of radiology image labelled “data”	Segmentation deep network (Inf-net)	[96]

## Data Availability

Data analyzed in this study were a reanalysis of existing data, which are openly available at locations cited in the reference section.
